The article "Post-induction hypotension with remimazolam versus propofol in patients routinely administered angiotensin axis blockades: a randomized control trial" was published in 2023. Journal: BMC Anesthesiol.

# Post-induction hypotension with remimazolam versus propofol in patients routinely administered angiotensin axis blockades: a randomized control trial

**DOI:** 10.1186/s12871-023-02188-9

**Published:** 2023-06-22

**Authors:** Seung Woo Song, Sujin Kim, Ji-Hyoung Park, Yun Hyung Cho, Yeong-Gwan Jeon

**Affiliations:** 1 Department of Anesthesiology and Pain Medicine, Wonju College of Medicine, Yonsei University, Ilsan-Ro 20, Wonju-Si, Gangwon-Do 26426 Republic of Korea; 2 Department of Anesthesiology and Pain Medicine, Wonju Severance Christian Hospital, Wonju-Si, Gangwon-Do South Korea

**Keywords:** Remimazolam, Hypotension, Anesthesia, Intraoperative care, Angiotensin-converting enzyme inhibitors, Angiotensin receptor antagonists

## Abstract

**Background:**

Certain routine medication could result in post-induction hypotension (PIH), such as angiotensin axis blockades, which are frequently administered as a first-line therapy against hypertension. Remimazolam is reportedly associated with lesser intraoperative hypotension than propofol. This study compared the overall incidence of PIH following remimazolam or propofol administration in patients managed by angiotensin axis blockades.

**Methods:**

This single-blind, parallel-group, randomized control trial was conducted in a tertiary university hospital in South Korea. Patients undergoing surgery with general anesthesia were considered for enrollment if the inclusion criteria were met: administration of an angiotensin converting enzyme inhibitor or angiotensin receptor blocker, 19 to 65 years old, American Society of Anesthesiologists physical status classification ≤ III, and no involvement in other clinical trials.

The primary outcome was the overall incidence of PIH, defined as a mean blood pressure (MBP) < 65 mmHg or decrease by ≥ 30% of the baseline MBP. The time points of measurement were baseline, just before the initial intubation attempt, and 1, 5, 10, and 15 min following intubation. The heart rate, systolic and diastolic blood pressures, and bispectral index were also recorded.

Groups P and R included patients administered propofol and remimazolam, respectively, as an induction agent.

**Results:**

A total of 81 patients were analyzed, of the 82 randomized patients. PIH was less frequent in group R than group P (62.5% versus 82.9%; t value 4.27, *P* = 0.04, adjusted odds ratio = 0.32 [95% confidence interval 0.10–0.99]). The decrease in the MBP from baseline was 9.6 mmHg lesser in group R than in group P before the initial intubation attempt (95% confidence interval 3.3–15.9). A similar trend was observed for systolic and diastolic blood pressures. No severe adverse events were observed in either group.

The article "Post-induction hypotension with remimazolam versus propofol in patients routinely administered angiotensin axis blockades: a randomized control trial" was published in 2023. Journal: BMC Anesthesiol.

**Conclusion:**

Remimazolam results in less frequent PIH than propofol in patients undergoing routine administration of angiotensin axis blockades.

**Trial registration:**

This trial was retrospectively registered on Clinical Research Information Service (CRIS), Republic of Korea (KCT0007488). Registration date: 30/06/2022.

## Introduction

General anesthesia induction is frequently followed by hypotension, namely post-induction hypotension (PIH), which is reportedly 18–50% [1–4]. The risk factors for hypotension following the induction of anesthesia include the regimen of induction, age, routine medications, such as angiotensin receptor blockers (ARBs) or angiotensin-converting enzyme inhibitors (ACEIs), and medical comorbidities of the patient [1, 2, 5]. Avoidance of intraoperative hypotension is highly recommended, since it is strongly associated with increased complications and 30-day mortality [6, 7].

Propofol is the most commonly administered agent for the induction of general anesthesia [8, 9]. However, the administration of propofol induces hypotension, mainly owing to reduced vascular resistance [1, 10]. In recent studies, remimazolam has been reported to be associated with lesser hypotension than propofol. Patients routinely administered angiotensin axis blockades could be more vulnerable to intraoperative hypotension [3].

Angiotensin axis blockades are widely administered in the surgical population, owing to their use as first-line treatment for hypertension. Adoption of an appropriate hypnotic agent is warranted to minimize hypotension and prevent potential complications in these patients. Therefore, we conducted a randomized controlled trial to compare the incidence of post-induction hypotension induced by remimazolam versus propofol in patients routinely administered angiotensin axis blockades.

## Methods

### Study setting

This study was designed as a single-blind, parallel-group, randomized controlled trial. The study was reviewed and approved by the Institutional Review Board of Wonju Severance Christian Hospital (CR321057; approval date: 20/07/2021) and registered with the Clinical Research Information Service of Korea (KCT0007488; registration date: 30/06/2022). This study was conducted in a tertiary university hospital in Wonju, Republic of Korea. This study was reported in compliance with the Consolidated Standards of Reporting Trials guidelines [11].

### Variables and assessments

The primary outcome was the incidence of hypotension following anesthesia induction. Hypotension was defined as a mean blood pressure (MBP) reduced 30% or more from the baseline MBP value or MBP < 65 mmHg, the threshold at which vital organ dysfunction can be initiated [6, 7].

The article "Post-induction hypotension with remimazolam versus propofol in patients routinely administered angiotensin axis blockades: a randomized control trial" was published in 2023. Journal: BMC Anesthesiol.

Blood pressure was recorded six times during anesthesia. Time points T0, T1, T2, T3, T4 and T5, were baseline, immediately before the first attempt of intubation, a minute after intubation, 5 min after intubation, 10 min after intubation, and 15 min after intubation, respectively. In case of the arterial cannulation is present, real-time arterial blood pressure values were recorded. Otherwise, blood pressure was monitored using the oscillatory method through a pneumatic cuff at the area of the brachial artery. The MBP measured using this method is widely validated and considered reliable when measured under proper conditions [12].

The secondary outcomes were heart rate, mean, systolic, and diastolic blood pressure (MBP, SBP, and DBP), and bispectral index (BIS). These variables were measured from T0 to T5. An attending anesthesiologist assessed and recorded the primary outcomes and intraoperative variables. These data were verified by the corresponding author upon a reviewing the anesthesia records.

### Participants

Patients undergoing surgery with general anesthesia were considered for enrollment if the inclusion criteria were met: routine administration of ACEI or ARB, 19 to 65 years old, American Society of Anesthesiologists physical status classification of III or lower, and no involvement in other prospective clinical trials. The exclusion criteria were as follows: emergency and outpatient surgery, a candidate for transfer to an intensive care unit, body mass index ≥ 35, uncontrolled hypertension (usual SBP > 160 mmHg) [13], pregnancy, breastfeeding, hepatic dysfunction of Child-Turcotte-Pugh Class C, and inability to understand the informed consent form. Withdrawal from the study was considered in case of anesthetic induction failure in spite of accordance with the protocol, hypersensitivity reaction during induction, and expression to discontinue participation in the study.

### Sample size

The incidence of hypotension was considered as 84% in the patients receiving angiotensin axis blockades and propofol as an induction agent based on a previous study [3]. An absolute difference of 30% or more was considered clinically significant. Upon setting an alpha value of 0.05 and a beta value of 0.2, 37 participants were required for each group. Finally, 41 patients were allocated to each group, reserving 10% of the withdrawals.

### Protocol

Assessment of eligibility and enrollment in the study was performed by the corresponding author. The participants were informed about the study via an informed consent form the day before the surgery, and provided sufficient time to determine their participation and sign the form. The participants were randomly assigned (1:1) to the propofol or remimazolam groups, namely groups P and R, respectively, using a sealed envelope system. A random allocation sequence was generated in advance by one of the authors (SWS) using R software. Paper cards containing the group allocations were sealed in opaque envelopes. Each sealed envelope was opened by another author (SK), and the patient notified the group allocation to an attending anesthesiologist 30 min before surgery. No anesthetic premedication was administered to the participants. The routine administration of ACEI or ARB was continued on the day of surgery.

The article "Post-induction hypotension with remimazolam versus propofol in patients routinely administered angiotensin axis blockades: a randomized control trial" was published in 2023. Journal: BMC Anesthesiol.

The induction drug was drawn in the anesthesia preparation room and the syringe was placed in a metal tin box. The patient and surgeon were blinded to the bolus drug administered by placing an opaque plastic cardboard, and blinding was maintained until the discharge of the patient from the post-anesthetic care unit.

The baseline blood pressure, heart rate, pulse oximetry, and BIS (BIS Complete Monitoring system, Covidien Ireland Limited, Dublin, Ireland) were recorded following the patient identification process. Other standard anesthetic monitoring devices, such as electrocardiograms, were also applied. Remifentanil infusion was initiated at a rate of 0.25 µg*kg^−1^*min^−1^. The patient was preoxygenated for two minutes. In group P, propofol 2 mg per kg ideal body weight (IBW) mixed with lidocaine 20 mg was injected following preoxygenation. Remimazolam was infused at the rate of 0.1 mg/h for blinding. In group R, normal saline 0.2 mL per kg IBW was administered and remimazolam was infused at a rate of 6 mg*kg^−1^*h^−1^ initially.

After loss of consciousness, remimazolam was infused at a rate of 1 mg*kg^−1^*h^−1^ in both groups. The infusion rate of remimazolam was increased in increments of 0.1 mg*kg^−1^*hr^−1^, up to the 2 mg*kg^−1^*hr^−1^ for BIS higher than 60. Rocuronium 0.8 mg/kg IBW was administered for neuromuscular block, and orotracheal intubation was attempted two and half minutes later. The BIS was maintained in the range of 40–60. Ephedrine 6 mg or phenylephrine 50 µg was administered if MBP reduced 30% or more from the baseline MBP value or MBP < 65 mmHg.

An additional bolus of rocuronium 0.15 mg/kg IBW was administered in cases of decreased pulmonary compliance or discretion of the surgeon. Fentanyl 1 µg/kg and ramosetron 0.3 mg were administered for postoperative pain control and postoperative nausea and vomiting prophylaxis.

### Statistical analysis

IBM SPSS 26 Statistics for Windows (IBM Corp., Armonk, NY, USA) was used for statistical analysis, and R Statistics 4.2.2 (R Core Team, Vienna, Austria) was used for visualization. The chi-square test was performed to analyze the primary outcome. The unadjusted and adjusted odds ratio of remimazolam versus propofol for the incidence of hypotension was calculated by logistic regression analysis, and the covariates were the administration of the drugs causing angiotensin axis blockade on the day of surgery and type of surgery.

The article "Post-induction hypotension with remimazolam versus propofol in patients routinely administered angiotensin axis blockades: a randomized control trial" was published in 2023. Journal: BMC Anesthesiol.

Decrease in the MBP, SBP, and DBP (blood pressure values subtracted from the baseline values) at T1 to T5 were compared using the t-test with Bonferroni correction to correct the multiplicity of the comparisons. The BIS and heart rate at T0 to T5 were compared using the t-test with Bonferroni correction. Other continuous variables were compared using the t-test, and categorical variables were compared using the chi-square test. Statistical significance was set as *P* < 0.05.

Blood pressure > 300 mmHg or < 30 mmHg and heart rate > 200 beats per minute were excluded from the analysis. Missing value analysis by SPSS revealed a few missing values (< 5%) in the total remifentanil dose and BIS values; however, they were randomly distributed. The missing values were excluded from the analysis.

## Results

From August 2021 to August 2022, 124 patients were assessed for eligibility and 82 patients were enrolled (Fig. 1). One patient in group R was withdrawn owing to variation in the airway management protocols; the surgical department required nasal intubation in this patient. A total of 81 patients were included in the final analysis.

**Fig. 1:** CONSORT Flow diagram

No significant differences were observed in the baseline characteristics between both groups (Table 1). Routine angiotensin axis blockades were administered as combination preparations with other antihypertensive drugs in 43 patients (53.1%). The participants fasted for 15.7 ± 4.3 h and the anesthesia time was 137.4 ± 72.5 min. The total dose of remifentanil was 1190.9 ± 733.5 µg.

**Table 1:** Baseline characteristics

	Propofol (*n* = 41)	Remimazolam (*n* = 40)
Age, y	60.1 ± 5.2	58.6 ± 6.4
Male, n (%)	28 (68.3)	25 (62.5)
Body mass index, kg/m^2^	26.3 ± 3.3	26.6 ± 4.0
Baseline mean blood pressure, mmHg	100.0 ± 11.0	99.4 ± 11.2
Baseline systolic blood pressure, mmHg	149.0 ± 19.7	146.0 ± 16.0
Baseline diastolic blood pressure, mmHg	82.6 ± 10.3	81.9 ± 11.5
ASA physical status classification, n (%)		
II	29 (70.7)	23 (57.5)
III	12 (29.3)	17 (42.5)
Administration of angiotensin axis blockade on the day of surgery, n (%)	37 (90.2)	37 (92.5)
Combination antihypertensive drugs, n (%)	25 (61.0)	18 (45.0)
Duration of preoperative fasting, h	16.1 ± 5.3	15.4 ± 3.0
Total time of anesthesia, min	150.9 ± 82.6	123.5 ± 58.2
Remifentanil dose, µg	1147.3 ± 749.9	1235.6 ± 723.6
Intra-arterial blood pressure monitoring, n (%)	3 (7.3)	4 (10.0)
Type of surgery, n		
Urology	11	15
General surgery	10	7
Otorhinolaryngology	6	5
Gynecology	4	5
Orthopedics	4	3
Others	6	5

There were no significant differences in the baseline characteristics

*ASA* American Society of Anesthesiology

The blood pressure decreased following the administration of induction agents in both groups (Fig. 2). The blood pressure increased following placement of the endotracheal tube and decreased again. The overall incidence of hypotension following general anesthesia induction was 72.8%. A total of 16 (19.8%), 13 (16.0%), 16 (19.8%), and 14 (17.3%) patients had hypotension at T1, T2, T3, and T4, respectively.

The article "Post-induction hypotension with remimazolam versus propofol in patients routinely administered angiotensin axis blockades: a randomized control trial" was published in 2023. Journal: BMC Anesthesiol.

**Fig. 2:** Mean blood pressure at each time point. MBP, Mean blood pressure. Bonferroni correction was done. *P < 0.008

The incidence of hypotension was not affected by the sex, age, or preoperative fasting time of the patients. Hypotension was less frequent in the patients administered remimazolam as the induction drug (62.5% vs. 82.9%; t = 4.27, *P* = 0.04). The absolute difference of hypotension was 20.4%, and the unadjusted odds ratio of incidence of hypotension was 0.34 (95% confidence interval [CI] 0.12–0.97). The adjusted odds ratio according to the type of surgery and administration of angiotensin axis blockade was 0.32 (95% CI 0.10–0.99). Specifically, MBP, SBP, and DBP decreased more abruptly in group P than in group R immediately before the intubation attempt (Table 2).

**Table 2:** Blood pressure reduction from the baseline at each time point and mean differences between the groups

		ΔBP_T1_	ΔBP_T2_	ΔBP_T3_	ΔBP_T4_	ΔBP_T5_
MBP	Propofol	30.0 ± 14.5 *	10.5 ± 22.8	27.8 ± 13.3	29.8 ± 10.3	29.4 ± 11.9
	Remimazolam	20.4 ± 13.9	12.0 ± 18.9	23.5 ± 13.6	26.7 ± 10.1	24.2 ± 11.9
	Mean differences (95% CI)	9.6 (3.3–15.9)	-1.5 (-10.8–7.7)	4.3 (-1.7–10.2)	3.1 (-1.4–7.6)	5.2 (0.0–10.5)
SBP	Propofol	51.1 ± 25.5 *	26.6 ± 36.3	50.7 ± 23.0	54.3 ± 18.3	52.1 ± 21.2
	Remimazolam	34.9 ± 22.4	25.7 ± 28.4	42.5 ± 20.6	46.1 ± 17.2	43.6 ± 20.6
	Mean differences (95% CI)	16.3 (5.6–26.9)	0.9 (-13.6–15.3)	8.2 (-1.5–17.8)	8.3 (0.4–16.1)	8.5 (-0.7–17.8)
DBP	Propofol	22.5 ± 12.2 *	5.1 ± 20.0	20.3 ± 13.3	21.2 ± 10.0	21.0 ± 11.4
	Remimazolam	14.5 ± 12.8	7.2 ± 17.7	16.8 ± 14.0	19.7 ± 11.4	16.8 ± 10.7
	Mean differences (95% CI)	8.0 (2.5–13.6)	-2.1 (-10.4–6.3)	3.5 (-2.5–9.5)	1.5 (-3.2–6.2)	4.2 (-0.7–9.2)

ΔBP, decrease in the BP at each time point; T1, T2, T3, T4 and T5, were baseline, immediately before the first attempt of intubation, a minute after intubation, 5 min after intubation, 10 min after intubation, and 15 min after intubation, respectively; *CI* confidence interval, *MBP* Mean blood pressure, *SBP* systolic blood pressure, *DBP* diastolic blood pressure

^*^P < 0.01; Bonferroni correction was applied for each variable

The heart rate was generally comparable between the two groups at every point of measurement (Fig. 3). One patient in group P had tachycardia (147 beats per minute) and demonstrated normal heart rate recovery through the administration of esmolol 10 mg. Another patient in the same group had hypertension (230/120 mmHg) a minute after intubation and was treated with nicardipine 500 µg.

The article "Post-induction hypotension with remimazolam versus propofol in patients routinely administered angiotensin axis blockades: a randomized control trial" was published in 2023. Journal: BMC Anesthesiol.

**Fig. 3:** Heart rate and bispectral index at each time point. Bonferroni correction was done. *P < 0.008

Flumazenil 0.5 mg was administered to one patient in group R owing to delayed emergence. The BIS was higher at five and ten minutes following intubation in group R than in group P (Mean differences 7.17 and 5.67, 95% CI of differences 2.81–11.53 and 0.87–10.47, respectively). No other adverse events were observed.

## Discussion

A remarkable proportion of patients (> 70%) in this study developed hypotension. This is higher than the general population and supports the finding that the patients routinely administered angiotensin axis blockades are vulnerable to PIH [2, 14]. PIH can be a remarkable risk factor for postoperative complications such as mechanical ventilation and extended length of stay [14, 15]. The causes of PIH are multifactorial, and various measures can be incorporated to prevent PIH, such as circulatory volume optimization, vasopressor administration, and arrhythmia correction [16]. Adopting remimazolam as an alternative hypnotic to propofol can be one of the measures to prevent PIH [17].

In cases of intraoperative hypotension, the amount of reduction in the blood pressure is also critical [18, 19]. A greater absolute maximum decrease in the mean arterial blood pressure resulted in a higher odds ratio of major adverse cardiac or cerebrovascular events in a previous multicenter retrospective cohort study; the odds ratio was 1.17 and 1.26 in the patients whose MBP dropped below 65 mmHg and 55 mmHg, respectively [18]. Since remimazolam administration resulted in a lower blood pressure reduction of approximately 10 mmHg than that of propofol in our study, less postoperative complications could be anticipated in patients administered drugs causing angiotensin axis blockade [20].

Another benefit of remimazolam as an induction agent is that the drug has the antagonist. There are some cases where rapid recovery after loss of consciousness is required. One example is difficult airway management. According to the multiple airway management guidelines, emergence and recovery of spontaneous ventilation are warranted in cases of supraglottic airway or endotracheal tube placement fails, but oxygenation is still possible [21–23]. The hypnosis induced by remimazolam is easily reversed with flumazenil in a minute if needed; therefore, remimazolam could be useful in patients undergoing difficult airway management with cardiovascular vulnerability [24].

The article "Post-induction hypotension with remimazolam versus propofol in patients routinely administered angiotensin axis blockades: a randomized control trial" was published in 2023. Journal: BMC Anesthesiol.

A trend of higher BIS was observed in participants administered remimazolam than in those who were administered propofol. Previous studies have reported a discrepancy between the BIS and sedative state in patients administered remimazolam [20, 25]. This is owing to the intrinsic limitation of the BIS, which is primarily better correlated with the hypnotic state induced by propofol than other anesthetic drugs [26]. However, no recall was instituted despite the higher BIS in previous studies [13, 27].

Our study has certain limitations. First, due to the loading dose of remimazolam in group R, the effect-site concentration after the loss of consciousness could be higher in group R. Further study adopting a target-controlled infusion model is required to overcome this limitation. Second, generalizability is limited due to the exclusion of high-risk surgical populations who require preparation for intensive care units. In addition, long-term postoperative outcomes, such as 30-day mortality, have not been studied. Further well-designed studies addressing the long-term postoperative impact of intraoperative hypotension in patients administered ARB or ACEI are warranted.

## Conclusion

Patients routinely administered angiotensin axis blockades are vulnerable to hypotension. Remimazolam results in lesser blood pressure reduction and lower instances of frequent PIH than propofol.

## Data Availability

The datasets used and analyzed during the current study are available from the corresponding author upon reasonable request.
